# Healthcare Engineering: A Lean Management Approach

**DOI:** 10.1155/2020/8875902

**Published:** 2020-10-03

**Authors:** Abdallah A. Abdallah

**Affiliations:** School of Applied Technical Sciences, The German Jordanian University, Amman, Jordan

## Abstract

This work tries to answer the following question: can healthcare be engineered using lean management tools? Lean is known to achieve successful results when implemented in the manufacturing sector. Typical results are operational cost reduction, cycle time reduction, and higher customer satisfaction. The service sector, however, has seen mixed results. For the last two decades, educators and healthcare professionals are trying to implement lean tools in healthcare. Some reported success and many did not, for variety of reasons. In this paper, we search the literature and reveal the special nature of healthcare services, success factors, and barriers facing implementation of lean in healthcare. We then conduct a survey of 18 elite Jordanian hospitals to study the case holistically. Statistical analysis of the survey results confirmed some of what the literature revealed; organizational leadership seems to be the most dominant factor, followed by knowledge of employees about lean, training, and patient satisfaction (customer focus). Another important finding, not captured by the literature, is that lean implementation success depends on educating physicians about continuous improvement and lean and ensuring they are part of the improvement team. Based on the revealed enablers and obstacles, we created a full lean implementation framework. This framework was then used along with selected engineering tools to implement lean in a major hospital successfully. Implementation results showed 60% of reduction in cycle time, 80% reduction in operational cost, and many other benefits.

## 1. Introduction

In a highly competitive world, all industrial and service sectors work relentlessly to save cost and enhance market standing. Healthcare organizations face even more challenges in keeping up with the competition and the cost of providing medical services. Delivering a high-quality medical service at an acceptable cost is the objective of owners and managers [1]. Many organizations used quality initiatives to achieve this challenging objective, but the journey is not always successful [2–4].

Healthcare professionals used various lean tools for the last two decades [5–7]. Many organizations were able to achieve some success in reducing cost, minimizing errors and improving profitability [8], but success is not always the result of lean implementation. Actually, lean implementation in healthcare has seen mixed success results; Barnabè et al. [9] declared that actual impact of lean is still a puzzle, since some see success with it and some do not. Similar notion is seen in the literature [10–12].

Kovacevic et al. [13] declared that many healthcare organizations used lean successfully and many others failed. Those who succeeded were able to see improvements in forms of saving time, saving walking distance, saving operational cost.

Mannon [14] showed how systematic use of lean in an integrated healthcare delivery system in Wisconsin (five hospitals and 27 physician clinics) changed the role of quality management from a system that was reactive to crises and quality issues to one that proactively pursues methods, processes, and strategies to improve quality for patients. Similarly, Aij [15] showed the importance of the role of leadership in providing successful implementation of lean in healthcare organization.

Typical lean studies try to run current operations with less human efforts, less space, less amounts of raw materials, and less cycle time [16]. Salam and Khan [17] showed how to implement lean successfully using a simulation-based lean management and implemented it in a private healthcare facility in Thailand. Their work resulted in higher efficiency by providing a better, faster, and safer healthcare system, which contributed to improved patient satisfaction. Kanamori et al. [18] studied the implementation of simple lean tools such as 5S (sort, straighten, shine, standardize, and sustain) for one year in Swedish health centres. The 5S program created changes in the work environment, including fewer unwanted items, improved orderliness, and improved labelling and directional indicators of service units. These efforts led to noticeable improvements in the quality of services provided.

Many researchers focused on the nature of healthcare systems and its interaction with any implemented methodology; Machado et al. [19] worked with two Brazilian hospitals in an exploratory study to see the possibility of implementing lean successfully. Their findings reveal that, unlike manufacturing, healthcare has a complex nature and needs a balanced approach to implement lean successfully. Fillingham [20] studied healthcare organizations in the UK and showed that healthcare sector is not ready for lean and resists it. Similar notion can be found in [21].

Radnor et al. [22] showed that lean is typically designed to be capacity-led, and hence there is limited ability to influence demand or make full use of freed up resources. Their findings showed that lean is indeed context-dependent and each implementation needs to address the individualized organizational culture. Manos et al. [23] showed that lean implementation has a success chance wherever we can achieve quick wins. Teich and Faddoul [24] argued that success is possible when we focus on the concept of “essential few” and customer value.

Poksinska et al. [25] studied healthcare services in Sweden and discovered that lean healthcare projects primarily target efficiency and little attention is paid to the patient's perspective. The study showed no significantly better results in patient satisfaction for primary care centres working with lean healthcare compared with those not working with lean. Furthermore, care centres working with lean showed no significant improvement in patient satisfaction over time. The authors believe that a holistic approach may provide better results when implementing lean in healthcare.

Some researchers studied the reasons behind implementation failure. A good literature review on implementation barriers and enablers can be found by Leite et al. [26]. The authors claim that 70% of lean projects fail in healthcare organizations. Similarly, Hussain and Malik [27] showed that the full deployment of lean principles was reported to be as low as 4% for the United States hospitals with 53% of the hospitals reporting only some level of lean implementation (according to studies performed by American Society for Quality—ASQ in 2009). Costa and Godinho Filho [28] claimed that the most important reason behind implementation failure is the lack of knowledge of lean management practices. Finally, Patri and Suresh [29] suggested that three factors could have the biggest impact on implementation success or failure: leadership, having a clear goal in advance for lean projects, and adequate training of the workforce.

D'Andreamatteo et al. [5] investigated lean implementation over 15 years in the USA. Their comprehensive literature review concluded that lean results appear to be promising, but scholars need to explore further the potential and the weaknesses of lean especially that every hospital represents a special case with a unique culture. Guillebaud [30] and Bateman et al. [31] showed similar conclusions and declared that, despite the rich literature, only a few papers addressed an entire organizational approach and very few studies are done in the Middle East. Similar findings can be found in [32].

This research consists of two phases. In the first phase, we create and distribute a survey designed to reveal reasons for success and failure of engineering and lean initiatives. In the second phase, we use knowledge gained thus far to create a framework that ensures implementation success. We then implement the framework in a major Jordanian hospital as pilot study to prove findings.

Throughout this work, we will focus on lean's effects on financial gains and patient satisfaction. Financial gains are achieved by saving money or adding income. Lean saves money when it leads to reduced cycle time, reduced raw material used, less quality issues, and less number of workers needed to do the job. Lean helps healthcare organizations to add income whenever it results into saving space or enhancing capacity to deal with more patients. Patient satisfaction is achieved by providing faster and effective service at a reasonable cost. We use the “customer focus” concept in this paper to highlight efforts that lead to patient satisfaction.

While both measures are tracked separately, they are really connected through focusing on quality. By decreasing cycle time and resources needed and by simplifying the process, we are really improving the speed and effectiveness of service, thus improving the patient satisfaction.

## 2. Methods and Research Model

### 2.1. Problem Statement

The healthcare industry continuously searches for new ideas to enhance the performance and improve financial standing. In this report, we study the effect of lean implementation on healthcare.

While lean practices are proven to create successful improvements in manufacturing environments, it does not have the same effect in the healthcare industry. In fact, over the last two decades, some healthcare organization saw some levels of success with lean implementation, and some did not.

The questions this research tries to answer are as follows:

- Can healthcare be engineered using lean management tools?
- What are the factors that support lean implementation and what are factors that hinder lean implementation in healthcare settings?
- What can be done to ensure successful implementation of lean in healthcare organizations?

### 2.2. Methodology

To answer the three questions listed in our problem statement, we start by summarizing the literature areas regarding lean implementation in healthcare.  Table 1 reveals the literature summary. From the reviewed literature, many implementation success factors, enablers, and barriers are revealed. These factors include upper management commitment or good leadership, active employee involvement, customer focus, holistic implementation approach, employee training, and external factors.

The listed literature is supported by countless research that can be found in specialized research databases such as PubMed under areas or subareas in Table 1 or under general search criteria such as lean healthcare [1, 5, 10, 11].

It is obvious that, under certain managerial scenarios, success is possible. To identify best environment for success, a structured survey was distributed and answered by 60 representatives working in 18 hospitals. The survey was answered by nurses, administrative personnel, physicians, and quality managers. The survey was designed to test multiple hypotheses according to the research model set forth. The hypotheses used in the model are as follows:

  H1: good leadership practices have a positive impact on lean implementation success and will lead to financial gains
  H2: good leadership practices have a positive impact on lean implementation success and will lead to patient satisfaction
  H3: employee involvement has a positive impact on lean implementation success and will lead to financial gains
  H4: employee involvement has a positive impact on lean implementation success and will lead to patient satisfaction
  H5: customer focus has a positive impact on lean implementation success and will lead to financial gains
  H6: customer focus has a positive impact on lean implementation success and will lead to patient satisfaction
  H7: external forces have a positive impact on lean implementation success and will lead to financial gains
  H8: external forces have a positive impact on lean implementation success and will lead to patient satisfaction
  H9: employee training has a positive impact on lean implementation success and will lead to financial gains
  H10: employee training has a positive impact on lean implementation success and will lead to patient satisfaction
  H11: holistic implementation approach has a positive impact on lean implementation success and will lead to financial gains
  H12: holistic implementation approach has a positive impact on lean implementation success and will lead to patient satisfaction

These relationships can be seen in Figure 1. Notice that implementation success is represented by performing well financially and improving patient satisfaction levels.

The six factors used in the survey were selected from the listed literature and were selected tested against good management sense. The healthcare industry, just like any other service, thrives on these six soft factors. Prior to running the surveys, interviews with management and quality professionals in all 18 hospitals indicated reasons for implementation failure. All the indicated reasons were related to these six factors. This is in line with the literature.

The six independent factors for implementation success are elaborated as follows: good leadership practices refer to full support and follow-up during implementation. Good leadership practices include coaching, mentoring, and authorizing needed training.

Employee involvement here focusses on involvement of physicians, since nurses and administrative staff are typically involved in any initiative, and their involvement is linked directly to the success of lean implementation in many published research papers. Physicians involvement, however, are not studied as much.

Customer focus refers to the level of interest in customer satisfaction in every change made in the healthcare organization. Most changes are made for the sake of minimizing operational cost or maximizing profit. This, however, may come at delays or less quality of services provided to the customer. A company with high customer focus thinks about the level of service provided to the customers as well as quality of services.

External forces refer to the pressure healthcare organizations face from the market. Competitive pressure and local regulations may cause the healthcare organization to look for initiatives that cut cost in every possible way. This, however, may hinder implementation success.

Finally, holistic approach refers to applying lean fully, not just one simple tool or just in one department. Applying an initiative holistically means taking into considerations all organizational and individual related factors and issues.

To ensure credibility of results, all healthcare organizations involved in this research were picked based on the following criteria:

- Involved in lean implementation or used lean tools for at least one year
- Have reports of performance measurements before and after implementation
- Mature enough and has been in business for at least 5 years
- The respondent has been involved in performance management or performance improvement for at least 3 years.

The criteria are set to guarantee seriousness of implementation in these organizations.

#### 2.2.1. Engineering and Lean Tools

As mentioned Introduction, this work includes two phases, and the second phase includes two parts: part one cares about creating a framework to guide successful implementation. This framework is built based on our findings from the literature and the survey results. In part two, we implement lean in a major Jordanian hospital using a collection of engineering tools.

From the literature review, one may be able to conclude that lean tools can be used in a healthcare facility to minimize cost, enhance patient care and patient satisfaction, speed up the healthcare process, etc.

The following lean tools can be used effectively in healthcare organizations:

5S (sort, straighten, shine, standardize, and sustain): 5S tools aim at making the working place clean, orderly, and free of clutter. Such tool builds great working ethics and reveals a clean operation. Healthcare organizations should always use 5S all the time as it represents a good fit with healthcare processes and objectives.
Visual management: The working place should be very visible. Every mistake is seen clearly. Inventories are exposed. Good work is seen to all. This can be achieved by using visual aids. Visual management tries to provide work related information to anyone without asking an employee, without using a computer or holding a meeting. This can be achieved by using colored signs, warning lights, instructional signs, painted floors, etc.
The seven harmful wastes: according to Womack and Jones [16], wastes in any system can be typically categorized as follows:
  - Waiting: employee or equipment idle time
  - Transportation: any movement that does not add value
  - Overprocessing itself: doing more work than necessary
  - Motion: wasted walking or movement
  - Poor quality: errors or rework
  - Inventory: storing excess inventory of anything
  - Overproduction: producing more, sooner, faster than required by the next step in the process
Reduction of these wastes in healthcare settings leads to faster service, less mistakes, and less cost.
Standardized work: standardized work stands for performing each process with the least cost, least number of steps, and best possible outcome. This can be achieved by establishing a continuous improvement process in place and by utilizing other lean tools such as *quality circles* and *suggestion systems*.
Value stream mapping (VSM): value stream maps are used to draw the process from the patient point of view. These maps reveal the seven wastes and help making the process better.
Load balancing: most healthcare organizations see imbalanced work loading, most of the time. Some departments are swamped with work while others do not have as much workload. Utilization of healthcare workers should be balanced. Lean utilizes most of the tools mentioned thus far to balance the load among departments and ensures a smooth flow of work.
In this research, we use a combination of engineering tools along with lean tools. Such tools can be of help to make the transformation to lean effective. Many engineering tools can be used, including the following:
Prioritization tools: many prioritization tools can be used including *Pareto chart* and *prioritization matrixes*. These tools are typically used to give priorities to areas of improvements, so that we work on some areas before others. They can also be used to categorize and prioritize problem causes.
Root cause analysis tools: many tools can be used to arrive to the root cause of a problem, including *brainstorming*, *fishbone diagram*, *benchmarking*, and *force filed analysis*. Such tools are powerful when used in combination with lean tools.
Simulation: simulation is used to represent the process, represents changes in the process, and performs “what-if “analysis. In this research, we use Arena® software to perform simulation.
Performance evaluation tools:at the end of each improvement project, performance improvements need to be quantified, measured, and presented. In this research, we propose using an index that quantifies the improvement in cost, cycle time, customer satisfaction, and quality improvement. The performance improvement index (PII) can be calculated as follows:

(1) $$\begin{array}{c} \text{PII}=\text{CI}*\text{CTI}*\text{CSI}*\text{QI,} \end{array}$$

where CI represents improvements in operational cost, CTI represents improvements in cycle time, CSI represents improvements in customer satisfaction, and QI represents improvements in quality performance.

Each of the four quantities is assigned a value of 1, 5, or 10. A value of 1 means no improvement. A value of 5 means good improvement and a value of 10 means great improvement. So, for any improvement project, if we do not expect a change in customer satisfaction because of this project, then CSI = 1. If this project causes great cost savings (say more than 50% of the current cost), then CI = 10. Similarly, if the quality is expected to improved and mistakes will be reduced by a good fraction, then QI = 5. Finally, if we expect cycle time to also decreased by a good fraction (no more than 50%), then CTI = 5. As a result, PII = 1 *∗* 10 *∗* 5 *∗* 5 = 250.

It can be noticed that PII will get values between 1 and 10000 and that the higher the value of PII, the better the indicator we get for quality initiative success.

## 3. Survey Analysis and Results

Initial sample included all governmental hospitals and 25 private hospitals in Jordan, with a total number of 31 hospitals. Initial number of survey respondents was 105. Introductory interviews that lasted two weeks revealed that only 18 hospital and 66 respondents are eligible to take the survey, based on eligibility criteria set forth. In the real sampling phase, only 60 healthcare professionals responded with answered surveys, which include 13 major questions with multiple branch for each question. Surveys and interview lasted for a total of four week.

The sample consists of 15 physicians with managerial posts in their hospitals, 23 nurses currently assigned administrative roles, 9 laboratory technicians currently assigned administrative roles, and 13 quality managers. All respondents were selected because they run some administrative tasks at their hospital, and they have been involved with performance improvement initiatives for at least two years.

The sample size is considered representative since participating hospitals represent all hospitals in the country with lean implementation experience.

All questions were close type and has a five-point Likert scale for each branch of each question, where 1 = totally disagree and 5 = totally agree.

The sample consists of 15 physicians, 23 nurses, 9 technicians, and 13 quality management professionals. All respondents have been involved with performance improvement initiatives for at least two years.

The survey consists of four parts: the first part collects personal information about those filling the survey. The second part includes questions that ensure lean implementation at the hospital. The third part includes questions about the six indicators shown in Figure 1. Finally, the fourth part asks about the level of financial improvements and patient satisfaction levels.

Statistical analysis and instrument validity used in this research is similar to those used by Salhieh and Abdallah [48]. The methodology used was designed and executed in a manner that ensures valid results. Face and content validity were ensured through summarizing the literature and testing each variable against professional knowledge and experience of each interviewee. Selecting healthcare professional from various backgrounds such as nursing, medicine, and management staff ensured internal validity of the study. Also selecting 18 different hospitals in different regions ensured external validity of the results. 90% of the interviewed managers agreed with the research model design. Each member of the sample was interviewed prior to filling the survey to ensure good knowledge of the research details.

Construct validity was performed as per Hair et al. [49] by performing exploratory factor analysis (EFA) and confirmatory factor analysis (CFA). Both EFA and CFA ensure unilateral effect of each construct in the model. Researchers [49, 50] suggested that eigenvalues for each construct to be more than 1 and a loading factor to be more than 0.4. Analysis revealed eigenvalues between 1.5 and 6.83 with all factor loading values greater than 0.4.

As seen in Table 2, all items have loading more than 0.60, which means all elements are effectives. Furthermore, the variance value of more than 0.5 suggests important influence of each independent variable on the behaviour of the two dependent variables [48]. The value of the variance is an initial indicator on the amount of effect. EFA and CFA not only provided validity of the analysis, but also revealed a strong causal relationship between selected dependent and independent variables. No cross loading is suspected based on the EFA-CFA analysis [49, 50].

CFA performs multiple statistical calculations and benchmarks each value of such statistics to a benchmark value. Each benchmark represents a standard, and if all benchmarks fit the standards, the model is said to be fit. First statistic is standard deviation of all effect in the model to be more than 0.5 [48]. A construct reliability score needs to be least 0.7 [49]. Also, according to Schreiber et al. [50] and Hair et al. [49], the *χ*^2^ value to degrees of freedom needs to be less than five. Tucker–Lewis index (TLI) and comparative fit index (CFI) needs to be greater or equal to 0.95. Finally, root-mean-squared error of approximation needs to be less than 0.06.

The calculated CFA values are all listed in Table 2, and CFA results with adequate goodness of fit and the model is, therefore, acceptable. All analyses have a statistical significance level of 1%.

The final step of analysis is to calculate the hypothesis significance. The goal is to create a model showing which independent factor has more effect on the results than other factors. The point here is to create a framework toward implementing lean successfully.

Results of hypothesis tests are shown in Table 3.

### 3.1. Discussion of Survey Results

From Table 2, we conclude that the most significant independent variables affecting the first dependent variable (financial gains) are “leadership,” “employee involvement,” and “using a holistic implementation approach,” while the most significant independent variables affecting the second dependent variable (patient satisfaction) are “leadership,” “employee involvement,” “customer focus,” and using a “holistic implementation approach.”

This is in line with many published literatures, with one exception: “employee involvement.” In this research, we used this term to highlight the role of physician involvement. Most published research focused on educating and involving nurses, laboratory technicians, and administrative staff but not physicians. This study found out that physicians could be great implementation assets or major obstacles. Educating physicians about lean and coaching them on their role can be a significant factor in successful implementation.

## 4. Framework for Successful Implementation

Since the outcome of lean implementation is not always success and those who succeed use certain success factors, it is clear that we have to create an implementation framework that provides high probability of success. Many researchers faced similar situation and came up with frameworks [1, 2, 14, 36]. Frameworks are not typically selected from other sources; they are rather created taking into consideration success factors and obstacles covered in each research.

Based on our findings so far, we concluded that lean can be implemented successfully in healthcare organizations, given that implementation follows a holistic implementation approach that uses success factors revealed from hypothesis testing. This approach is built into a framework as shown in Figure 2.

The framework consists of several steps as follows:

(1) Establish a need to improve financial standing or patient satisfaction: improvement initiatives such as lean are need-driven. If management does not see a major need for improvement in the financial performance or patient satisfaction levels, no support will be provided for lean implementation.
(2) Ensure upper management involvement and continuous support: once the need has been established, lean cannot survive without continuous support from upper management. Leadership influence here is a major factor. Involvement of upper management in performance reviews and implementation audit reviews is vital.
(3) Build a holistic implementation approach: this starts with understanding the culture and level of resistance for new initiatives and then, a good understanding of the internal environment for the organization with a focus on strengths and weaknesses points. The initiative will be implemented everywhere in the organization, and it is essential to start by establishing a good feeling of the as-is status.
(4) Perform internal marketing campaign to all employees to convince them on the new initiative: it is vital to tell everyone why we need lean? Why is it the way to prosper? What is their role? How did others become successful with it? Internal marketing campaign is performed through emails, portals, employee meetings, news leaflets, etc.
(5) Perform training for all and include physicians: after knowing the weaknesses, quick training need analysis (TNA) can be established. And, training programs should be performed to everyone as awareness sessions, while members of the lean team are offered specialized training.
(6) Select an implementation team: part of the holistic approach is the involvement of everyone; however, a small lean team will be responsible for implementation success and follow-up. This team should include nurses, physicians, laboratory technicians, and administrative staff.
(7) Train and empower the implementation team: the team has to have access to upper management. It has to have high visibility in the organization.
(8) Design an implementation approach: while the implementation is supposed to be holistic, implementation should start in areas where it will show highest success levels or quick wins. Expected values of PII for any initiative may help to select where to start, or we can just use any prioritization tool to select where to start. It helps to start implementing lean in areas of lowest expected resistance, but the plan should include all areas in the organization.
(9) As much as possible, use the following tools in this sequence:
  - 5S
  - Visual management
  - Eliminating the seven wastes
  - Simulation
  - Implementing standardized work
  - VSM
  - Load balancing
Also, as needed, use any of the root-cause analysis tools in any step.
(10) Audit implementation: one of the important failure reasons is the lack of follow-up. An annual audit plan needs to be set for all areas. The lean team will be responsible for auditing the implementation progress.
(11) Calculate PII and announce the results.
(12) Review and continuously improve: a quarter review (every three months) is suggested to take place between lean team and the upper management. The review will act as a tool to enhance audit results and to set continuous improvement plans. The review will highlight areas with high PII results and will set the stage for future improvement initiatives.

The framework is designed to ensure implementation success; it takes into consideration obstacles and enablers covered in the literature and the survey performed in this research. The design of the framework does not contradict with any literature known to the authors or listed in this work, but the value of the framework will not be quantified unless it is experimented on a real case study. The use of the framework has to show a positive impact on financial gains for the hospital, improved patient satisfaction, and most importantly better performance quality, which can be measured in less mistakes and more effective treatments.

## 5. Case Study

To test the findings of our survey and the framework, a major hospital (more than 250 beds and more than 1000 employee) was used as a case for this research. The hospital was selected for the following reasons:

- The hospital is accredited by JCI (Joint Commission International)
- Most processes are considered standardized since they have gone through cycles of improvements
- The hospital is ISO 9001 certified
- Upper management are always eager to use new improvement ideas

Steps 1 and 2 of the framework were not performed since upper management appreciates any improvement initiative. We began with step and decided to use the framework hospital-wide but to start by selecting areas with immediate need, as it will be shown next.

In step 4, we started a marketing campaign. The mission was not difficult since employees of the hospital are used to quality initiatives mandated by JCI and ISO 9001, but staff were not familiar with lean and its effectiveness in healthcare, so many marketing activities took place to tell everyone how well did some health organizations do with lean.

Next, we established a hospital-wide training program. The training was an introductory course in lean performed for everyone. The idea of the short training is to be informative and to tell people that everyone will be part of the movement. Next, we selected a team of 12 (3 physicians, and the rest are nurses and technicians). This team was trained for two weeks on lean and problem solving tools and tactics.

The real work starts in the next few steps. The team selected to work in the emergency room (ER) area for the following reasons:

- Two of the team members work in that area.
- ER has the highest number of complaints from customers.
- Most medical insurance issues are seen in the ER.
- ER has high density of employees (technicians, nurses, and physicians).
- Patients do not easily find their path once they arrive to the ER and tend to need guidance.
- ER has operation room, triage room, 10 beds, X-ray room, reception, accounting department, pharmacy, and lab. The utilization is not the same for each of these areas, and high imbalance can be seen.
- Operational cost is considered very high by management, since 10% of the payroll is related to ER. In addition, the overhead cost concerning the operations room, triage room, beds area, and the labs is about 20% of the hospital overhead cost.

A comprehensive review of using lean tools in ER can be found in [10, 51, 52].

The process in the emergency room is described by the flow chart in Figure 3. A quick look at the chart provides an idea about the amount of waiting and walking performed by every ER patient.

To fully understanding the process, a team of three technicians collected data for 7 days of full operation. The average waiting and walking distances taking place in the ER is shown in Table 4. The table shows that, on average, every patient spends 119 minutes inside the ER and walks 854 steps (almost 300 meters). These values are considered very high for an emergency patient.

To build the simulation model, we need two things: process flow (Figure 3) and a number of inputs such as patients' arrival time, task times, waiting times, and resource availability. A team of three technicians collected starting time (arrival time) and task time for each task. They also recorded duration of waiting time between steps for each patient and the number of resources working in each step. The collection of data lasted for 7 days. Each set of data is entered into Arena's input analyzer, and the software assigned the best distribution fit for each set of data. As an example, distribution of arrival data can be seen in Table 5. Arena provides best-fit distributions for all the data we collected.

The simulation model is ready to run after all process data is entered for the ER (Figure 4). The model is validated after that. Validation is performed by comparing model output with actual output. For example, is the model report of resource utilization match actual resource utilization? Is waiting time for resource in the model similar to that in reality? We keep modifying the model until we achieve at least 90% validation. After validation, the model is ready for what-if analysis. We can perform process changes and see how it affects all aspects of process performance.

The baseline model revealed that most of the process is spent in waiting or walking. The model also revealed high utilization rate for the nurses in the ER bed area and the X-ray but low utilization in other areas.

Finally, we created a value stream map for the process at the ER prior to make any improvements. The full map can be seen in Figure 5.

The VSM chart, while simple in nature, reveals that half the time spent by the patient in the ER is not adding any value; only 65 minutes are used to add value in this process, the remainder of his time is a form of waste.

### 5.1. Applying Lean and Engineering Tools

After collecting all needed data and information about the process in the ER, the team started brainstorming sessions with the following two goals:

1. Eliminate none value adding time as much as possible
2. Lower the total time for the ER experience to all patients

The length of the cycle time for patients in ER can be seen as a result of many reasons. A fishbone diagram was created by the team to reveal possible root causes and areas for improvement. The diagram is shown in Figure 6.

The following can be deducted from all the tools used so far:

- The layout of the ER does not help; patients walk too much inside the facility.
- Patients walk from one room to another aimlessly without a clear guide.
- The assignment of tasks for nurses and physicians is not done in any systematic manner.
- Some resources are highly utilized and some are not. This imbalance needs to be resolved.
- Some mistakes take place due to paper work and documents that flow in a none electronic manner.
- Patients spend good amount of time waiting for available resource.

Based on this holistic picture we created for the current process and the team is ready to use improvement tools.

The following were recorded as brainstormed ideas:

1. Since most of the interior building sections are made of Gibson boards, the medical observation room (where the beds are located) is suggested to be enlarged and some of the partitions that split it from the laboratories to be eliminated.
2. Since the medical observation room is now much bigger, the triage room can now have a door leading to the waiting room, which in turns leads to the medical observation room.
3. All the rooms will have visual aids and signs showing patients where to sit and where to go and what to do.
4. Eliminating the reception area: this area is currently staffed with two technicians who are swamped with miscellaneous, unorganized work. Instead, the team suggested naming one, well-trained technician or nurse as a joker (someone who can fit in many places). This joker will have two main jobs: (i) greet the patients as they come into the ER and guide them between steps (ii) assign tasks to all those working in the ER in a manner that guarantees smooth flow of patients.
5. Cross train employee (nurses and technicians) so that any employee can help other areas when needed and under the supervision of the joker.
6. Every area that has high level of work will push a button that flags a red light observed by the joker, so that he himself goes and helps or sends someone who does not have high load of work.
7. Merging some tasks for those who have low utilization: for instance, the lab technicians are now responsible for data entry of patients since they were found to have the least workload.
8. The process will be focused on two things: (i) no patients waiting for service and (ii) no empty bed in the observation room. These two items will be focus of the joker and will guarantee smooth flow of patients with minimal waiting.
9. Distributing employees in the ER so that patients always have a visible employee. This high customer exposure guarantees higher customer satisfaction and resolve customer issues swiftly and quickly.
10. Killing the majority of paper work: this can be done by adding computers in every area that has customer contact, such as triage room, medical observation room, pharmacy, lab, and X-ray. The nurse in the triage room establishes a new live page (file) for every patient that walks into the ER, and then any employee or physician who does anything to that patient enters what he performed and forwards his file to the next department. By the time the patient walks to the next department, he finds them ready for him, with little or no waiting. For Example, by the time he arrives to pharmacy, he finds his medications prepared and ready for pick up. The patient's file is closed by the accounting department.
11. Minimizing the possibility of any mistake (mistake proofing): this can be achieved by establishing controls in the computer program that prevent those who use the patient file from forwarding his file to the next department without going through the proper procedure. This is a simple programming matter.
12. Making the flow of patients (patient arrival ⟶ triage ⟶ observation room ⟶ lab ⟶ X-ray ⟶ pharmacy ⟶ accounting  department ⟶ patient departure) in a “U” shape. This can be achieved by ensuring the arrangement of these departments is in a sequence with a corridor in the middle. The “U” shape arrangement guarantees high visibility and allows all to serve the customer well and observes any problem as it happens.
13. The furthest department form ER is the X-ray room. The team suggested relocating it to a closer location, but this suggestion will take 4 months of implementation.
14. Simplifying the entire process: for example, the physician is considered a precious resource, so he is freed from doing all paper work, and this became the job of less utilized technicians. In addition, the joker became responsible for faster patient movement inside the facility. In addition, much of the paper work has been eliminated. In short, physicians, nurses, and technicians are more involved now in value-adding work.
15. Providing every patient with a simple card before he or she exits to ask him or her about their experience at the ER.
16. Eliminating all the clutter including all paperwork, all unneeded towels, and covers from the ER area.
17. Connecting the hospital warehouse with the ER through an automated request system, so that any time the ER needs supplies of anything, a request is pushed, and the warehouse supplies the department with its needs. This request system is made the responsibility of one of the technicians.

The above lean ideas were incorporated, and the current process was changed toward a faster service and better customer experience. These ideas are summarized in Table 6. The table clearly shows the impact on cycle time, walking distance, and customer satisfaction.

### 5.2. Simulation of Process Changes

After gaining approval for suggested process changes, all changes were incorporated in the original simulation model except relocating the X-ray room. The management asked that this change be delayed for future considerations.

Simulations model results revealed the following:

- The maximum employee utilization is 92%
- The minimum employee utilization is 67%
- The observation room bed utilization 73%
- Total average cycle time of patients in the ER is 33 minutes which is considered ideal in global standards.
- A decrease of number of employees working in the ER by 3 nurses and technicians.

Simulation produces these important performance results by randomly selecting values from the distribution of each input piece of data, then running the process in animated mode and observing each time how much each resource is idle or utilized, and how long each patient is waiting in the ER. This makes simulation a powerful tool to predict almost all process outputs once distributions are defined for input data.

A full week of data collection, after the changes took place, revealed that actual average time of patients in ER is 46 minutes, and the new total average walking distance is 406 steps, which is considered a great improvement from the old status.

The team enforced an audit process that guarantees proper implementation of all suggested improvements. In addition, a quarter review is set in place to be the upper management platform of follow-up.

## 6. Results and Discussion

The case hospital is an ideal candidate to perform the experiment of lean implementation since it has a leadership that is willing to try any initiative under the umbrella of continuous improvement. In addition, the most employees are trained on quality initiatives, which makes it even better.

All suggested ideas were implemented with the best possible efforts. The resulted new times and walking distance are shown in Table 7. The table shows great improvements form the old process.

In addition to improvements seen in cycle time and walking distances, ER saw a number of other benefits including the following:

(i) Minimizing all waiting times that lowers patient satisfaction.
(ii) Minimizing all types of walking in the ER.
(iii) Better customer experience and customer satisfaction. This was seen immediately through customer satisfaction cards that was added to the process and collected during a whole week after implementation.
(iv) Better quality performance and less mistakes. Mistake proofing of the process and the automation of all information flow reduced the mistakes by an average of 80% as seen in the measurements taken a week after lean implementation and comparing that week with historical data. Some of the mistakes that was eliminated or reduced include the following:
  - Misdiagnosis
  - Poor monitoring
  - Lab errors
  - Contaminated or misplaced test samples
(v) Operational cost was reduced by 55% due to the following:
  - Reduced number of employees by 3
  - Cycle time is now 60% less than it used to be
  - Capacity increase
  - Less mistakes and rework
  - Less paperwork and less material used

The 55% estimate is our first estimate based on one-week worth of work after the implementation. Estimate of cost savings included salary of 3 employees, estimation of all the paper and material saved, and the estimated time spent performing rework.

This estimate is in line with simulation output and is expected to be firmed up after the first few quarter reviews:

- Better employee skills. Employees are now more empowered and loyal.
- Higher level of pride among employees.

We can easily calculate PII according to the following equation:

(2) $$\begin{array}{c} \text{PII}=\text{CI}*\text{CTI}*\text{CSI}*\text{QI,} \end{array}$$

where CI = 10 since cost improvement is more than 50%, CTI = 10 since cycle time improvement is more than 50%, CSI = 5 since we can feel improvement in customer satisfaction but we cannot tell yet if the improvement exceeded 50%, and QI = 10 since quality improvement exceeded 50%

As a result,

(3) $$\begin{array}{c} \text{PII}=5000\text{.} \end{array}$$

This is a great result, and this project will be used as a benchmark inside the case hospital as they plan for similar performance improvements in many areas especially the warehouse, operations rooms, etc.

## 7. Conclusions and Future Work

While the manufacturing sector has been enjoying benefits of lean implementation for decades, effective implementation in healthcare organization is not easy but achievable. Taking into consideration internal and external forces and thinking holistically is vital, a smart implementation strategy has to be designed to overcome implementation obstacles.

This research agrees with the literature on the importance of leadership and support of upper management, but an important finding of this research is the role of physicians in lean implementation. They can be a major obstacle if not involved in a proper manner.

This paper shows that implementation success in healthcare can be achieved similar to that in the manufacturing industry, but the service nature of healthcare organizations needs to be taken into consideration. Once a good understanding of internal environment is created, a proper holistic approach can be implemented. Continuous follow-up is the final requirement for implementation success.

The case hospital revealed how easy implementation becomes when the upper management is on board, but if this is not the case, then following the proposed framework guarantees success, even if it takes longer.

The use of PII as a measure of success is necessary, since it quantifies performance improvements, and it can be used to show various levels of success in different areas in each organization.

The most important conclusion is the answer to the main question in this research: yes, healthcare can be engineered to be lean, by following the proposed framework.

Future work can focus more on the role of physicians. How can they be a driving force in such initiatives? And how can they enhance follow-up and continuous improvement efforts?

Future work can also extend the findings of this research and the implementation framework to other quality initiatives, by using the proposed framework including the use of PII and simulation. This is in line with recently published research in other quality initiatives such as six sigma [53], balanced scorecard [54, 55], and business process management [56, 57].

Future work can link lean implementation success with accreditation and internal culture; culture of accredited healthcare organization may be different from that of unaccredited organizations, but is this a factor in implementation success? A question to be answered by future research.

Finally, future work can extend the fruitful finding of this research to policy makers who are responsible for healthcare management. Lean tools, especially 5S, visual management, and standardization should become standard procedures at all healthcare institutions. Policy-makers can also limit the maximum time and maximum walking distances for patients, especially ER patients.

## 8. Research Limitations

This research was proven by a case study in a large accredited hospital. Results may vary in smaller size hospitals. Smaller hospitals are run with limited number of employees and tend to scrutinize every operational cost more than large hospital. Future research may test the model used in this research in hospitals with less than 50 beds.

Another category of hospitals that was not studied in this research is the unaccredited hospitals category. Unaccredited hospitals do not have the same operational standards of accredited hospitals and may not value lean management in the same manner.

The case and survey was implemented in Jordan, where physicians have great administrative power. Physicians were included in the survey and in the research team. In different countries, physicians may have limited administrative power; therefore, their participation may not be needed in such surveys.

Future research can tackle these research limitations.

## Figures and Tables

**Figure 1:** Research model.

**Figure 2:** Proposed implementation framework.

**Figure 3:** Flow chart for the process at the ER.

**Figure 4:** Initial simulation model for the process at the ER.

**Figure 5:** VSM for the process at the ER.

**Figure 6:** Fishbone diagram for the long cycle time at the ER.

**Table 1:** Summary of literature review on lean implementation.

Area of research	Subarea	Authors	
*Key implementation success factors*	Leadership skills and involvement	Achanga et al. [33]	Kundu and Manohar [34]
		Aij [15]	Maijala et al. [35]
		Doss and Orr [36]	Najem et al. [37]
		Hamid [38]	Steed [39]
		Kumar et al. [40]	Vermaak [41]
	Holistic implementation of lean	Bateman et al. [31]	Machado et al. [19]
		Costa and Godinho Filho [28]	Parkhi and Suresh [29]
		Guillebaud [30]	Poksinska et al. [25]
	Employee involvement	Hamid [38]	
		Harmon et al. [42]	Vermaak [41]
	Organizational culture	Achanga et al. [33]	
		Hamid [38]	Kundu and Manohar [34]
		Kumar et al. [40]	Najem et al. [37]
	Customer focus	Hamid [38]	Kumar et al. [40]

*Implementations benefits achieved*	Waste reduction, customer satisfaction, cycle time reduction, administrative benefits, employee satisfaction, better performance quality, etc.	Folinas and Faruna [43]	Papadopoulas [44]
		Graban [8]	Rexhepi and Shrestha [45]
		Kanamori et al. [18]	Shazali at al. [46]
		Hussain and Malik [27]	Womack and Jones [16]

*Enabelers and barriers*		Bateman et al. [31]	Manos et al. [20]
		Costa and Godinho Filho [28]	Patri and Suresh [29]
		Fillingham [20]	Radnor et al. [22]
		Leite et al. [26]	Teich and Faddoul [24]

*Success implementations*		Aij [15]	
		Kovacevic et al. [13]	Mannon [14]

*Failed implementations*		Fillingham [20]	Øvretveit [3]
		Nembhard [4]	Shortell et al. [2]

*Mixed results*		Barnabè et al. [9]	Maijala et al. [35]
		D'Andreamatteo at al. [5]	Rees and Gauld [11]
		de Souza [12]	Savage et al. [10]

*Implementation framework*		Costa and Godinho Filho [28]	Hussain and Malik [27]
		Dahlgaard et al. [47]	Shazali at al. [46]

**Table 2:** EFA and CFA analyses.

	Standardized loading	Eigenvalues	*t* values (all significant to *p* < 0.000)	Construct reliability	Average variance extracted
Leadership		6.83		0.877	0.815
Financial gains	0.712		32.621		
Patient satisfaction	0.623		28.442		
Employee involvement		3.11		0.790	0.786
Financial gains	0.802		17.348		
Patient satisfaction	0.703		21.622		
Customer focus		5.54		0.755	0.722
Financial gains	0.669		11.655		
Patient satisfaction	0.813		17.278		
External forces		1.50		0.686	0.568
Financial gains	0.724		8.546		
Patient satisfaction	0.821		5.629		
Employee training		4.95		0.823	0.788
Financial gains	0.771		15.243		
Patient satisfaction	0.728		18.418		
Holistic approach		6.13		0.884	0.803
Financial gains	0.690		30.326		
Patient satisfaction	0.825		25.621		

	Goodness of fit indicators: *χ*^2^ (12) = 26.22 (*p* < 0.001) ⟶ ratio *χ*^2^ to df = 2.383 *(criterion: <5)* Tucker–Lewis index = 0.981 *(criterion: ≥0.950)* Comparative fit index = 0.967 *(criterion: ≥0.950)* Root-mean-squared error of approximation = 0.042 *(criterion: <0.06)*				

**Table 3:** Hypotheses testing calculations.

Hypothesis	*p* value (0.0000)	Conclusion
Leadership		
H1	1.2	Very significant
H2	3.5	Very significant

Employee involvement		
H3	19.3	Very significant
H4	22.1	Very significant

Customer focus		
H5	46.2	Significant
H6	16.9	Very significant

External forces		
H7	70	Significant
H8	96	Marginal

Employee training		
H9	55.9	Significant
H10	41.3	Significant

Holistic approach		
H11	12.6	Very significant
H12	9.8	Very significant

**Table 4:** Average time and walking distance in the ER.

Task	Walking (steps)	Time (min)
Patient arrival	30	1
Check vital signs in triage room		5
Fill out patient history		2
Wait for empty bed	36	14
Nurse inspects patient	20	4
Wait for physician		10
Full check		7
X-ray	380	13
Lab	174	25
Wait for physician		10
Diagnosis		3
Walk to pharmacy	98	5
Pick up prescription		10
Payment collection	106	5
Check out	10	5
Total	854	119

**Table 5:** Probability distribution for patients' interarrival times.

Patient arrival	Shift A	Shift B	Shift C
Time	8:00–15:00	15:00–22:00	22:00–8:00
Distribution	Exponential	Exponential	Exponential
Mean	2.36	2.17	7.79
Chi-squared test	0.58	0.75	0.29
Result	Do not reject	Do not reject	Do not reject

**Table 6:** Lean ideas in the case hospital.

Idea number	Lean tool	Benefits
1	Waste reduction (waiting and movement)	Walking and waiting reduction Smooth flow of patients
2	Waste reduction (waiting and movement)	Walking and waiting reduction Smooth flow of patients
3	Visual management	Better customer satisfaction
4	Process standardization Waste reduction (unnecessary process)	Process simplification Faster processing better customer satisfaction
5	Employee empowerment	Process simplification Faster processing better customer satisfaction
6	Process flow Load balancing	Faster processing better customer satisfaction More satisfied employees
7	Process flow Load balancing	Faster processing better customer satisfaction More satisfied employees
8	Process flow Elimination of waiting waste	Faster processing better customer satisfaction
9	Process flow	Better customer satisfaction Faster process
10	5S	Better customer satisfaction Faster process
11	Mistake proofing	Better customer satisfaction
12	5S Visual management Process flow	Better customer satisfaction Faster process
13	Eliminating movement waste	Faster process
14	5S Eliminating over processing waste	Faster process
15	Customer focus	Better customer satisfaction
16	5S Eliminating rework waste	Faster process
17	5S	Faster process

**Table 7:** Average time and walking distance in the ER after lean implementation.

Task	Walking (steps)	Time (min)
Patient arrival	25	1
Check vital signs in triage room		5
Fill out patient history		2
Wait for empty bed	17	1
Nurse inspects patient	15	3
Wait for physician		1
Full check		5
X-ray	235	10
Lab	35	10
Wait for physician		1
Diagnosis		1
Walk to pharmacy	51	2
Pick up prescription		1
Payment collection	18	3
Check out	10	
Total	406	46

## Data Availability

For the sensitivity of interviews, many of the organizations surveyed asked not to disclose any of the data used. As a result, data used to support the findings of this study are confidential and cannot be made available.

## Acronyms

5S: Five words starts with the letter “S.” Each word represents an action under lean management umbrella. The five words are sort, straighten, shine, standardize, and sustain
CFA: Confirmatory factor analysis, a statistical tool used to ensure analysis validity
CFI: Comparative fit index, a statistical tool used to ensure analysis validity
CI: Improvements in operational cost after implementing a new initiative
CTI: Improvements in cycle time after implementing a new initiative
CSI: Improvements in customer satisfaction after implementing a new initiative
VSM: Value stream mapping, a method to draw the process in lean management
EFA: Exploratory factor analysis, a statistical tool used to ensure analysis validity
ER: Emergency room
JCI: Joint Commission International
PII: Performance improvement index
QI: Improvements in quality performance after implementing a new initiative
TLI: Tucker–Lewis index, a statistical tool used to ensure analysis validity
TNA: Training need analysis.
